# Designing of SiO_2_ mesoporous nanoparticles loaded with mometasone furoate for potential nasal drug delivery: *Ex vivo* evaluation and determination of pro-inflammatory interferon and interleukin mRNA expression

**DOI:** 10.3389/fcell.2022.1026477

**Published:** 2023-01-06

**Authors:** Yasir Mehmood, Hira Shahid, Kashif Barkat, Muhammad Ibraheem, Humayun Riaz, Syed Faisal Badshah, Hitesh Chopra, Rohit Sharma, Eugenie Nepovimova, Kamil Kuca, Martin Valis, Talha Bin Emran

**Affiliations:** ^1^ Riphah Institute of Pharmaceutical Sciences (RIPS), Riphah International University Faisalabad, Faisalabad, Pakistan; ^2^ Saffron Pharmaceuticals (Pvt.) Ltd., Faisalabad, Pakistan; ^3^ Department of Pharmacology, Faculty of Pharmaceutical Sciences, Government College University Faisalabad, Faisalabad, Pakistan; ^4^ Faculty of Pharmacy, University of Lahore, Lahore, Pakistan; ^5^ Rashid Latif College of Pharmacy, Rashid Latif Khan University, Lahore, Pakistan; ^6^ Chitkara College of Pharmacy, Chitkara University, Chandigarh, Punjab, India; ^7^ Department of Rasa Shastra and Bhaishajya Kalpana, Faculty of Ayurveda, Institute of Medical Sciences, Banaras Hindu University, Varanasi, Uttar Pradesh, India; ^8^ Department of Chemistry, Faculty of Science, University of Hradec Králové, Hradec Králové, Czechia; ^9^ Neurology Clinic, University Hospital, Hradec Králové, Czechia; ^10^ Biomedical Research Center, University Hospital Hradec Kralove, Hradec Králové, Czechia; ^11^ Department of Neurology, Charles University in Prague, Faculty of Medicine in Hradec Králové and University Hospital, Hradec Králové, Czechia; ^12^ Department of Pharmacy, BGC Trust University Bangladesh, Chittagong, Bangladesh; ^13^ Department of Pharmacy, Faculty of Allied Health Sciences, Daffodil International University, Dhaka, Bangladesh

**Keywords:** drug delivery, nasal spray, controlled release, *ex vivo* study, mesoporous silica nanoparticles

## Abstract

The main objective of the current research work was to synthesize mesoporous silica nanoparticles for controlled delivery of mometasone furoate for potential nasal delivery. The optimized sol–gel method was used for the synthesis of mesoporous silica nanoparticles. Synthesized nanoparticles were processed through Zeta sizer, SEM, TEM, FTIR, TGA, DSC, XRD, and BET analysis for structural characterization. The *in vitro* dissolution test was performed for the inclusion compound, while the Franz diffusion experiment was performed for permeability of formulation. For the determination of expression levels of anti-inflammatory cytokines IL-4 and IL-5, RNA extraction, reverse transcription, and polymerase chain reaction (RT-PCR) were performed. The MTT assay was also performed to determine cell viability. Synthesized and functionalized mesoporous silica nanoparticles showed controlled release of drugs. FT-IR spectroscopy confirmed the presence of the corresponding functional groups of drugs within mesoporous silica nanoparticles. Zeta sizer and thermal analysis confirmed the delivery system was in nano size and thermally stable. Moreover, a highly porous system was observed during SEM and TEM evaluation, and further it was confirmed by BET analysis. Greater cellular uptake with improved permeability characteristics was also observed. As compared to the crystalline drug, a significant improvement in the dissolution rate was observed. It was concluded that stable mesoporous silica nanoparticles with significant porosity were synthesized, efficiently delivering the loaded drug without any toxic effect.

## 1 Introduction

Chronic rhinosinusitis (CRS) is a prevalent inflammatory condition which affects the nasal cavity and paranasal sinuses. These disturbing conditions may significantly disrupt a person’s daily functioning and quality of life (Soyka et al., 2012). Nasal congestion and discharge are associated with this inflammatory condition which may last for at least 12 weeks. Combination of surgical and medical treatments is the most preferred therapeutic strategy for individuals suffering from CRS, whereas the use of topical and systemic steroids is also considered a cornerstone for therapy of this illness. Endoscopic sinus surgery (ESS) is generally acknowledged as the invasive method for treating CRS, which is resistant to standard medicinal therapy since it enhances sinonasal airway potency and opens the sinuses, resulting in lowering the severity of the inflammation. Nevertheless, it is not always a straightforward and benign treatment, and possible risks include postoperative severe bleeding, mucosal adhesions, infection, inflammation, and poor surgical results. Steroids are often preferred for controlling CRS owing to their powerful anti-inflammatory characteristics. Although oral steroids are effective, their practice is accompanied with various side effects. Because of this, topical steroids are preferred owing to their good safety profile. Similarly, intranasal delivery through different nasal sprays is highly frequent and typically favored both by patients and clinicians. Intranasal steroids are an effective therapeutic technique of CRS therapy. Mometasone furoate (MF) has been found to be effective in managing nasal inflammatory diseases (Passali et al., 2016). It has been used in clinical practice for sinonasal purposes for more than 20 years, and considerable literature has proven its therapeutic characteristics for such disorders. However, MF is a highly lipophilic and poorly aqueous-soluble (0.0108 mg/ml) medication with a relatively low risk of systemic absorption. Bioavailability has been reported as <1%, while trials of recurrent doses of inhaled corticosteroids show a bioavailability of 11%. An inhaled dosage has a terminal half-life of about 5 h. So there is a big challenge to make MF soluble and increase its bioavailability (Passali et al., 2016). There are a variety of excipients, including co-solvents, micellar solutions, surfactants, complexing agents, and lipid formulations, that may be used to improve the drug’s solubility and its bioavailability. Traditional drug delivery methods have limitations; however, these hurdles may be circumvented using nanotechnology-based drug delivery. Sub micrometer solid particles or nanoparticles (NPs) are capable of transporting a wide range of therapeutic agents, including peptides, nucleic acids, and tiny hydrophilic and hydrophobic moieties, to specific biological environments. Nanoparticles (NPs) have the potential to enhance medication stability and solubility and bioavailability at the site of action and duration of action *via* regulated release. Nanoparticles have an emerging application because of their unique chemical, physical, and biological properties (Singh et al., 2020a). There are many types of nanoparticles and techniques to manufacture it. However, among them, mesoporous silica nanoparticles (MSNs) have been widely and extensively used as controlled drug delivery systems (DDS) throughout the last decade (Wang, 2009). Mesoporous silica materials are attractive for a number of reasons, including their enormous surface area, inertness, malleability in terms of volume and pore size, and amenability to functionalization related to chemical nature (Chen et al., 2004; Cao et al., 2009; Kilpeläinen et al., 2009). In addition, nanoparticles may induce specific physiological responses in target cells and tissues without triggering any unintended side effects (Bhattacharya et al., 2022). Nanoparticle-modified chemicals have shown improved medication delivery and tissue targeting (Chopra et al., 2021). It is sometimes challenging to get the appropriate therapeutic benefits with conventional drug delivery methods, but these alternatives may assist (Chopra et al., 2022). All of these features allow for more precise management of medication loading and release. Precise regulation of pore size, shape, particle size, and pore geometry is crucial for biological uses. The overall pore size and orientation is established by composition of the surfactant templates. The size and morphology of the MSNs may be adjusted from spherical to rod or worm-shaped by adjusting the molar ratio of silica precursors and surfactants or solvents. The inclusion of base catalysts (Cai et al., 2001; Lin and Mou, 2002) and organic swelling agents or co-solvents (Kresge et al., 1992; Anderson et al., 1998) and the incorporation of organoalkoxysilane precursors throughout the co-condensation process all have a role in determining the final particle size (Huh et al., 2003). This research aimed to improve solubility and regulate drug release by creating MSNs laden with a poorly aqueous soluble drug (MF), and it can be delivered through a nasal spray. Nano-sized particles (particle diameter 200 nm) were prepared using the sol–gel method, and after drug loading, surface functionalization with APTES was performed. SEM, TEM, BET, XRD, FT-IR, DSC, and TGA were used to examine their physicochemical properties in depth (Salonen et al., 2005; Heikkilä et al., 2007; Yang et al., 2008; Kapoor et al., 2009). After preparation of MSNs loaded with MF and functionalized with APTES, these were used to prepare the nasal spray.

## 2 Materials and methods

### 2.1 Chemicals

Cetyltrimethylammonium bromide (CTAB), tetraethyl orthosilicate (TEOS), 3-aminopropyl triethoxysilane (APTES), acetonitrile, and hydrochloric acid were purchased from Dae-Jung chemicals (Gyeonggi, Korea). Saffron Pharmaceuticals (Faisalabad, Pakistan) donated mometasone furoate. Dialysis membranes having molecular weight cutoff (MWCO) of 8,000 Da were acquired from Spectrum Medical Industries (Houston, Texas, United States). Double-distilled water prepared in the Pharmaceutics Research Laboratory of the Faculty of Pharmacy, University of Lahore, was used throughout the experiments. Reagents and solvents which were used during the experiment were of analytical grade and were used as received.

### 2.2 Syntheses of mesoporous silica nanoparticles (MSNs)

Synthesis of mesoporous silica nanoparticles using a modified sol–gel approach has been recently described by our group (Mehmood et al., 2019). MSNs produced with a ratio of acetonitrile to water as 1:1 were chosen for this investigation after much trial and error in our prior research. Specifically, a 250-ml flask was used to combine 100 ml of acetonitrile and water (1:1) at 35°C for 15 min. The aforementioned solution was then added to 300 mg of CTAB while being continuously stirred at the same temperature in a nitrogen environment. An hour after obtaining a clear solution, 5 ml TEOS as a silica precursor was gently added through a 10-ml syringe while the mixture was continuously stirred. Nearly instantly, the solution became opaque or milky white, an indication that a reaction had begun. Under nitrogen pressure, the white gel (MSNs) was filtered through a 0.1 Sartorius filter, cleaned by washing three times with deionized water, and dried in a desiccator at 25°C for one night. The bulk was then dried and calcined at 500°C for 6 h to eliminate any remaining surfactant template.

### 2.3 Functionalization of mesoporous silica nanoparticles

Fabricated MSN-MF was functionalized with 3-aminopropyl triethoxysilane (APTES) groups by optimizing a post-fabrication method. For this purpose, a three-necked flask was taken and 100 mg MSN-MF was added to it. The entire reaction system was purged with nitrogen. After purging with nitrogen, 2.0 ml APTES in 50 ml aqueous solution was added, and refluxing of the system was carried out at 70°C under nitrogen with continuous stirring for 10 h (Zhang et al., 2010a; Wang et al., 2016). The final product was filtered and washed several times with ethanol and then dried at 90°C overnight (Zhang et al., 2010a). The samples were labeled as MSN-MF.

### 2.4 Preparation of nasal spray nano formulation by using mometasone furoate-loaded MSNs

Nasal spray formulation was prepared by using already mometasone furoate-loaded MSNs (MSN-MF). In this preparation, we have used the same excipient (microcrystalline cellulose) as an innovator. Stability and drug leakage were studied under accelerated conditions.

### 2.5 Characterization of functionalization

#### 2.5.1 Ninhydrin assay

Amino group presence on the surface of silica particles may be detected using a ninhydrin reagent test. The formation of the ninhydrin–amino complex is confirmed by the presence of a purple color in the reaction mixture, which indicates that ninhydrin has reacted with the amino group on the silica particles (Araghi and Entezari, 2015). Acetate buffer and a ninhydrin solution (3%) were prepared in water and ethanol (50/50) (Lu, 2013). Then, 100 mg of MSN-MF was taken and mixed into 10 ml of the ninhydrin solution. After 15 min, stay color was formed, and it was further diluted with water and its absorbance was checked on 570 nm wavelengths using a UV–visible spectrometer (Shimadzu 1,600 equipment), which was also confirmed by the FT-IR study.

#### 2.5.2 Determination of entrapment efficiency

About 100 mg of MSN-MF was separately weighed. Around 100 ml of methanol was taken, and the weighed quantity of MSN-MF was separately mixed with it with continuous stirring for 1 h. The mixture was filtered after 1 h of continuous stirring, and the filtrate thus obtained was quantified for MF using a validated HPLC method. A 1000 pump with an attached UV–Vis detector (Japan) was the structural alignment of the HPLC system (Shimadzu LC 20AB). An Agela C18 column (250 × 4.6 mm, 5 µm) was optimized and used as the stationary phase, whereas ammonium acetate buffer (pH = 7.6), methanol, and acetonitrile at a ratio of 10:50:40 (%v/v) were used as the mobile phase, respectively. The injection volume was 20 µl, flow of the mobile phase was maintained at a rate of 1.0 ml/min, while the wavelength of the UV detector was set at 254 nm. After processing, the obtained chromatograms were then compared with the standard, and the drug loading efficiency was calculated in triplicate.

$$Entrapment\;Efficiency\;\left(\%\right)=\frac{Drug\;added-Free\;drug}{Drug\;added}\;X\;100.$$ (1)

#### 2.5.3 Particle size and polydispersity index (PDI)

Determination of mean particle size, PDI, and zeta potential was carried out by photon correlation spectroscopy (PCS) by optimizing the particle size analyzer (Zetasizer, Malvern Instruments, United Kingdom). The nano-nasal spray was prepared using filtered water, and then it was immediately used to determine the particle diameter and PDI.

#### 2.5.4 FT-IR spectroscopy

The FT-IR spectrometer equipped with an attenuated total reflection crystal cell and designed by Thermo Scientific Nicolet iN5 FTIR, United States, was used to carry out the FTIR spectroscopic study. A small amount of the sample was added to the instrument with the help of a spatula. Using this method, optimizing the range of 400–4,000 cm^−1^, spectra of MSN, MF, poloxamer, MSN-MF, and nano-nasal spray were recorded.

#### 2.5.5 Differential scanning calorimetry study (DSC)

A differential scanning calorimetry study (DSC) of pure drugs, MSN, and MSN-MF was performed by using Diamond Series DSC designed by Perkin Elmer, United States. The samples were scanned under nitrogen atmosphere at a rate of 10°C min^−1^ with a temperature range of 30–300°C after being loaded into standard empty aluminum crucibles pierced with holes in the center.

#### 2.5.6 X-ray powder diffraction study (XRPD)

An X-ray powder diffraction study (XRPD) of pure drugs, MSN, and MSN-MF was performed by an X-ray powder diffraction analyzer, designed by D8 ADVANCE, Bruker, Germany. The radiation used was cobalt-filtered Fe^2+^ with a wavelength of 1.7890°A.

#### 2.5.7 Morphology study

Scanning electron microscopy (SEM) (JEOL Ltd, Tokyo, Japan) was used for the morphological analysis. MSN crystals of the pure drug and MSN-MF were mounted onto metal stubs having a dual-sided adhesive tape coated with gold by using a sputter coater.

#### 2.5.8 Nitrogen adsorption–desorption analysis

Nitrogen adsorption–desorption analysis was used for determination of the surface area, pore volume, and size of blank and loaded MSNs. The Gemini VII 2390 surface area analyzer (Micromeritics Instrument Corp, Georgia, United States) was used for the study, operating at −196.15°C. Prior to analysis, the sample was degassed at 200°C for 24 h. The procedures of Barrett–Joyner–Halenda (BJH) and Brunauer–Emmett–Teller (BET) were applied on adsorption–desorption data in order to determine pore characteristics (Brunella et al., 2016).

#### 2.5.9 *In vitro* release study

*In vitro* released experiments using the dialysis membrane technique were performed on both the pure medication and the nano-nasal spray. One milligram of medication in the nano-nasal spray was injected into a dialysis bag (MWCO 12–14000 Da, Medicell International Ltd, 239 Liverpool Road, London) which was used to create a closed pouch-like structure. The dialysis bag loaded with the moieties was then suspended in two different medium solutions of 500 ml each: 0.1 M HCl with pH 1.2 and phosphate buffer solution with pH 7.4 with constant stirring at 37 ± 0.5°C and 50 rpm. Two milliliter (ml) samples were taken at regular intervals up to 8 h and were replaced with new media at the same volume and under the same conditions. The filtrate was then collected at a pore size of 0.45 m and diluted in the mobile phase for further HPLC analysis (Zhang et al., 2010b). The percentage of release was determined using the formula (2) (Khalid et al., 2018a; Barkat et al., 2018):

$$Drug\;release\;percentage=\frac{sample\;absorbance}{standard\;absorbance}\times 100.$$ (2)

#### 2.5.10 Kinetic modeling

The pattern of drug release during the dissolution study from formulation was calculated by applying different mathematical models to evaluate the behavior of the nano-nasal spray.

##### 2.5.10.1 Zero order

A zero-order approach is used to describe drug release from the nano-nasal spray. The following equation can be used to describe this approach (Khalid et al., 2018a).

$$Qt=Q_{o}+K_{o}t.$$ (3)

In the aforementioned equation, Q_t_ is the therapeutic agent quantity release within “t” time, whereas Q_0_ is the initial quantity of the therapeutic agent in formulation, and K_0_ is the rate constant.

##### 2.5.10.2 First order

The first-order kinetic model describes that release of the active moiety through nanoparticles depends upon the drug quantity in the formulation. It is described by following Eq. 4 (Barkat et al., 2017).

$$logC=\log C_{o}-\frac{kt}{2.303}$$ (4)

where C_0_ is the initial active moiety amount within nanoparticles and k is the first-order rate constant. −k/2.303 determines the slope.

##### 2.5.10.3 Higuchi model

The Higuchi model explains that drug release follows diffusion (Fick’s law) (Barkat et al., 2018). Release of the moieties from nanoparticles which follow Higuchi model release kinetics is mentioned in Eq. 5 (Khalid et al., 2018b).

$$Ft=K_{₂}\times t½1/2.$$ (5)

In the aforementioned equation, F_t_ describes the quantity of drug that remained undissolved, and K_2_ states the Higuchi rate constant.

##### 2.5.10.4 Korsmeyer–Peppas model

The Korsmeyer–Peppas model tool is used to describe the release of the active moiety being entrapped in a polymeric system. This model is expressed by the following equation (Barkat et al., 2018).

$$\frac{Mt}{M\infty }={\text{Kt}}^{n}.$$ (6)

In the aforementioned equation, Mt/M∞ depicts the therapeutic agent quantity liberated from the polymeric network system at “t” time. The term k in the aforementioned equation describes the model release rate constant. If n (diffusion exponent) ≤ 0.45 or 0.45 < n < 0.89, release of the therapeutic agent follows Fickian and non-Fickian diffusion, respectively. In another case when n = 0.89 or n > 0.89, release of the therapeutic agent follows the case-2 transport or super case-2 transport, respectively (Dash et al., 2010).

### 2.6 Statistical analysis

Particle size, PDI, and zeta potential values are expressed as mean ± SD. For the selection of significant model terms (factors) and the models, statistical analysis and goodness of fit statistical criteria (predicted and adjusted *R* ^2^, adequate precision) implemented in DX^®^ were used, respectively. The *p*-value <0.05 was considered significant.

### 2.7 Physical appearance, viscosity, and pH determination

The MSN-MF nano-nasal spray was checked for its physical properties. One percent dispersion prepared in the aqueous medium was tested for pH by using a digital pH meter (Ino lab WTW 730, United States). The formulated MSN-MF nano-nasal spray was evaluated for their viscosities at 0.5, 1, and 2 rpm by using the Brookfield viscometer (Model DV-II) using Spindle #21.

### 2.8 *In vitro* diffusion studies

The Franz diffusion cell was used during the experiment in which a silicon membrane was employed. Evaluation of the *in vitro* characteristics of MSN-MF nano-nasal spray and commercial nasal spray permeation was performed using a vertical Franz diffusion cell (SES Analytical Systems, GmbH, Germany) over a silicon membrane by having the donor surface area of 1.2 cm^2^ and a receptor volume of 5.2 ml. The Franz diffusion cell having epidermal side up consists of a semisynthetic membrane [silicon SAMCO (Nuneaton, United Kingdom)] inserted between its donor and receptor chambers. Paraffin-coated MSN-MF samples were placed in a donor chamber with a capacity of 1 ml. However, the water in the receptor chamber is a 7.4 pH phosphate buffer saline maintained at 37 ± 0.5°C. Half an hour before the experiment, at 37 ± 0.5°C, the membrane was in touch with the receptor phase. Over the course of 8 h (0.5, 1, 2, 4, 6, and 8 h), 0.5-ml samples were taken at regular intervals during the receptor phase and evaluated using a UV-spectrophotometer set to 254 nm, while the cell was refilled with an equal quantity of freshly produced buffer solution (Abdul et al., 2020; Thakur et al., 2020).

### 2.9 *In vitro* cell viability studies

The human hepatoma cell line (HepG2) was obtained from American Type Culture Collection (ATCC) (Manassas) which was grown by the University of Lahore. DMEM supplemented with 10% (v/v) FBS in a 95% (v/v) humidified atmosphere and 5% (v/v) CO_2_ at room temperature was used for optimization of the cells. A day before incubation with MSN-MF, the cells were seeded. For the measurement of succinate dehydrogenase mitochondrial activity as an indicator of cell viability/proliferation, the MTT (3-(4,5-dimethylthiazol-2-yl)-2,5-diphenyltetrazolium bromide) assay was used (Mosmann, 1983). The MSN-MF nano-nasal spray of different concentrations (50–400 μg/ml) was added to the cell medium for 24 h. After that, 15 μl of MTT was added to each well and incubated at 37°C for additional 4 h. The medium with MTT was then aspired carefully, and the formed formazan crystals in each well were solubilized in 100 μl of dimethyl sulfoxide (DMSO). Afterward, the absorbance of the dissolved formazan crystals was measured at 570 nm using a microplate reader (Patel et al., 2009). The percentage cell viability was determined using the following formula.

$$\%\;cell\;viability=\frac{Abs\;of\;treated\;cell-Abs\;of\;blank}{Abs\;of\;Control-Abs\;of\;Blank}X\;100.$$ (7)

### 2.10 Hemolytic investigations

To conduct the hemolytic study, blood was collected (rat blood) in an ethylene diamine tetra acetic acid-containing tube, centrifuged at 1,500 rpm for 5 min, and the supernatant was removed while the precipitate was washed three times with phosphate buffer saline (PBS). Around 200 μl of washed blood sediment was taken, and 3.8 ml of phosphate buffer saline was added and vortexed for few minutes. After that, these samples were kept at 37°C for 2 h, and the mixture was centrifuged for 5 min at 1,600 rpm. An absorbance of the supernatant at 541 nm was evaluated. In this experiment, Triton was selected as a positive control and phosphate buffer saline as a negative control. % hemolysis was determined by using Eq. 8.

$$\%\;Hemolysis=\frac{ABS\;sample-ABS\;blank}{ABS\;positive-ABS\;blank}\times 100\%.$$ (8)

### 2.11 Acute toxicity studies

According to the Organization for Economic Co-operation & Development Toxicity guidelines, the animal model was used for MSN-MF nano-nasal spray formulation toxicity. Six rats weighing 150–170 g were purchased from the Tollinton market, Lahore, Pakistan, and divided into two groups and kept in the animal house of Lahore University for 14 days. The MSN-MF nano-nasal spray was topically administered by nasal route in the test group surviving on water and food compared to the control group. On the 14th day of the study, blood samples were collected, and various biochemical parameters were examined (Erum et al., 2015).

### 2.12 Lung histopathology

Dissected lung tissues were fixed in buffered 10% formalin and dehydrated using varying amounts of ethanol for histopathological analysis. Sections of tissue 6 m thick were cut using a microtome after being immersed in paraffin wax. Hematoxylin and eosin (H&E) staining was then used to examine the infiltration of inflammatory cells into the isolated tissues. It was determined that goblet cells could be distinguished using a periodic acid–Schiff (PAS) stain. Inflammatory cell infiltration and goblet cell hyperplasia were two of the characteristics examined microscopically in the lungs.

### 2.13 Determination of pro-inflammatory cytokines IL-4 and IL-5 mRNA expression

Chemokines and cytokines have a mediating role in airway inflammation. Eosinophils, lymphocytes, and mast cells all generate cytokines. Allergic asthma is characterized by severe inflammation, which is mostly triggered by proinflammatory cytokines (IL-4 and IL-5), which are primarily generated by Th-2 cells. Th-2 lymphocytes, neutrophils, mast cells, and eosinophils may all be attracted by these proteins. Both eosinophils and mast cells play crucial roles in the development of asthma. Bronchoconstriction is caused by the cytokines and leukotrienes produced by these cells. The reverse transcription polymerase chain reaction was used to assess IL-4 and IL-5 mRNA expression levels in tissue. The TRIzol technique was used to extract total RNA from blood. The following was used to synthesize cDNA: 1 μl of oligo dt primer (10 M), 4 μl of 5X reaction buffer, 0.5 μl of RNAse inhibitor (20 U/L), 2 μl of dNTP mix (10 mM), 0.5 μl of M-MuLV enzyme (200 U/L), and nuclease-free water q. s to 20 μl. Templates consisted of 1,000 ng of total RNA per reaction. The resulting cDNA was frozen at −20°C for later use in the polymerase chain reaction. For the PCR, we combined 2 μl of cDNA, 0.75 μl of forward and reverse primers (10 M), 6 μl of PCR master mix, and 2.5 μl of nuclease-free water. A total of 35 cycles of denaturing at 95°C for 10 s, annealing at 58–60°C for 20 s, and elongating at 72°C for 30 s constitute a standard PCR technique. First, the PCR result was analyzed visually by running it on an agarose gel (2%), and then, using densitometry in an image editing program, it was partially quantified.

## 3 Results

Treatment of CRS, a chronic inflammatory illness defined by the buildup of highly viscoelastic mucus in the sinuses, often begins with the use of topical steroids. Poor distribution to the nose and sinuses is a common reason why topical steroid treatment fails to provide optimal therapeutic results. Mechanistically stable nanoparticles have the potential to enhance treatment outcomes by enabling more uniform drug distribution to specific areas, increased contact duration, localized drug elevation, and fewer systemic side effects. The improved sol–gel approach was used to synthesize MSN-MF. Adding MSN-MF to a nasal spray formulation led to the discovery that this was the optimal formulation for boosting solubility.

### 3.1 Drug entrapment efficiency

The results of the determined MF entrapment efficiency within MSN were very good. The results showed that the maximum MF entrapment efficiency percentages were obtained in the ratio of acetonitrile and water (1:1) at 35°C for 15 min. In this ratio, the maximum MF entrapment efficiency percentage was 41.00, and functionalization was approved by the ninhydrin test which showed the appearance of purple color, which was further confirmed by a UV–Visible spectrometer.

### 3.2 Particle size and polydispersity index (PDI)

Particle size and size distribution of this formulation were determined and characterized using DLS. Figure 1A shows a size distribution diagram of MSN-MF generated in water. The DLS result showed that the hydrodynamic diameter of MSN-MF was 200 nm, with PDI of 0.297 and −10.2 zeta potential. The result showed significant PDI of 0.297, which indicated good dispersions of particles.

**FIGURE 1:** Size distributions of the MSN-MF nano-nasal spray.

### 3.3 FT-IR analysis

For identification and characterization of functional groups present on the mesoporous silica particles, FT-IR spectroscopy in the region of 500–4,000 cm^−1^ was used. Absorption bands at 797.97, 1,053.78, 1,636.88, and 3,396.49 cm^−1^ were observed in mesoporous silica nanoparticles, which are often attributed to the siloxane bond (797.97) (Wardhani et al., 2017), Si–O–Si bending (1,053.78 cm^−1^), and the silanol (Si-OH) symmetric stretching (3396.49) (Sevimli and Yılmaz, 2012; Liu et al., 2015) and bending vibrations at 1636 cm^−1^ (Liu et al., 2015; Wardhani et al., 2017).

As shown in Figure 2, MF exhibits unique FT-IR spectra. The FT-IR characteristic absorption bands for MF were observed at 3,430 (O–H str.), 2,938, 2,886 (C–H str.), 1726 (C=O str. In ester), 1,658 (cyclic C=O str.), 1,610 (acyclic C=O str.), 1,468, 1,393 (C–H def.), and 1,026 cm^1^ (C–O str.). There are two carbonyl peaks between 1,650 and 1,750 cm^−1^, which correspond to the two carbonyl groups present in the MF molecule (Chen et al., 2005). At 1,635 cm^−1^, the existence of the amide-I group was indicated, and at 1,540 cm^−1^, the presence of the amide-II (N-H bend) group in MF was indicated, which was due to the stretching of C = O. The presence of a small peak at 1,350 cm^−1^ indicates the presence of a carboxylic group (38–40).

**FIGURE 2:** FT-IR analysis of MSN-MF, MSN-amine, MSN, MF, and commercial product.

FT-IR of MSN-MF presents low-intensity peaks that indicate successful loading of MF into MSN particles. Si–O–Si bending (1,053.7 8 cm^−1^) and silanol (Si–OH) symmetric stretching (3,396.49) (Sevimli and Yılmaz, 2012; Liu et al., 2015) and bending vibrations at 1,636 cm^−1^ (Liu et al., 2015; Wardhani et al., 2017) were present in MS-MF and MSN-MF nano-nasal spray, which clearly indicated the presence of MSN-MF in the stable form within the nasal spray. Major peaks were observed at 2,900 cm^−1^ and 1,710 cm^−1^ as shown in Figure 2, which indicated C–H str. Carbonyl bond formation by the amine group results in absorption at a lower wavenumber 1,706 cm^−1^. In FT-IR of MSN-MF, acyclic stretching (C=O) was moved from 1,610 cm^−1^ to 1,655 cm^−1^. Discrete bands were observed in the range of 970–1,215 cm^−1^ wavenumber because of amine functionalization.

### 3.4 Thermal analysis

A differential calorimeter model Q-2000 manufactured by TA United States, was used to evaluate MF, MSN, and MSN-MF. The temperature range was 25°C–500°C adjusted at a rate of heating 20°C/min. The response of MSN, MF, and MSN-MF formulation against heat flow is shown in Figure 3. As shown in Figure 3, the DSC curve of MSN exhibits an endothermic peak at 50°C, which corresponds to its intrinsic melting points due to dehydration and elimination of other volatile components. An exothermic peak at about 75°C is observed, which can be attributed to glass transition temperature T_g_. The MF differential scanning calorimetry graph is shown in Figure 3. Two overlapping endotherms were detected at approximately 233°C and 238°C followed by an exothermic reaction at 242°C. The presence of the complex thermal events around the melting point indicates significant degradation of MF during melting. Significant weight loss was detected over the same temperature range by TGA (Figure 3) (Chen et al., 2005).

**FIGURE 3:** Thermal analysis of MSN, MF, and MSN-MF.

In MSN-MF, no sharp exothermic peak was observed at 233°C and 238°C that recognized that MF is poured into pores of MSN in amorphous form. However, a weak and broad endothermic peak appears at 90 ℃ in MSN-MF, which indicates the non-crystalline state of drug entrapment into MSN. Over a temperature range of 70°C–120°C by TGA, 3.2% weight loss was observed. Figure 3 agrees with considered water content of 3.3% for the monohydrate. The melting peak depression of MSN-MF may be linked to partial interaction of drugs with the surface of mesoporous nanoparticles rich in silica groups, resulting in partial amorphization of MF drugs (Maleki and Hamidi, 2016).

### 3.5 Morphology analysis

Fabricated MSNs generally have high porosity. A spherical shape was observed when MSN particles were scanned under the electron microscope. The presence of the porous surface might be due to phase evaporation during hardening of the particle. The presence of the porous surface of MSN is an important feature in the delivery system for the controlled release characteristics of the entrapped drug moieties (Tiwari, 2016). Figure 4C shows the electron microscopic view (SEM and TEM) of MSN-MF, and the view showed well-dispersed MSN particles. API crystalline particles and commercial products of the nasal spray are also shown in Figure 4A, B (bright-field microscopy), which depicted large crystal particles within the formulation.

**FIGURE 4:** **(A,B)** Bright-field microscopy images of API **(A)** and commercial nasal spray **(B)**. **(C)**. TEM and SEM images of MSN-MF.

### 3.6 X-ray powder diffraction (XRPD)

The XRPD patterns for MF, MSN, and MSN-MF are presented in Figure 5. MF exits sharp peaks with crystalline forms (Chen et al., 2005). The XRD patterns were similar to those of polymorphs with major peaks observed at characteristic diffraction peaks that can be depicted at 2-theta values of 9.3, 9.7, 11.3, 13.8, 14.8, 16.0, 18.9, and 19.48 (Chen et al., 2005), corresponding to the crystalline trend of MF. However, no prominent peaks were noted in MSN-MF, which confirmed the shifting of MF into the amorphous form because of enlarged pore confinement with the polymer matrix.

**FIGURE 5:** XPRD patterns of pure MF, MSN, and MSN-MF.

### 3.7 Nitrogen adsorption–desorption analysis

MSN-MF synthesized by the modified sol–gel method has high porosity. BET analysis was used for the evaluation of the surface area, pore size, and volume of the unloaded drug and loaded drug MSN. From the results, a significant reduction in the BET surface area of MSN-MF was observed compared to that of the unloaded MSN due to the entrapped drug. Likewise, pore size and pore volume were also decreased in MSN-MF as compared to those of unloaded MSN shown in Figure 6.

**FIGURE 6:** Nitrogen adsorption/desorption isotherms of blank MSN and MSN-MF.

### 3.8 Physical characterization

For nasal spray applications, MSN-MF nano spray formulation was developed in liquid form. The pH of nano-nasal spray formulation was 6.1 (±0.1) according to USP, which is appropriate for nasal products. The viscosity of formulation was 89 cpi at 25°C. Nasal products are usually evaluated for mechanical properties in order to investigate their extrudability from the container and spreadability of the product. The spreadability of the formulation is related to its hardness and compressibility, while adhesive and cohesive properties of formulation have the ability to retain on the surface and regain the structure after application. In the present study, MSN-MF nano-nasal spray showed a minor increase in compressibility and hardness, with slight decrease in retaining time and reconstructing structure of MF.

### 3.9 *In vitro* transcellular permeability

The present study mainly aimed to check the *in vitro* transcellular permeability of formulated MSN-MF nano-nasal spray of pH 7.4 through a silica membrane. The de-aerated buffer was used to fill the clean dried receptor cell and was permeable for 15 min at 37°C in a heated magnetic block. The pre-hydrated silica membrane was used between the matched donor and receptor compartment, and the indoor compartment was filled with 1 g of MSN-MF nano-nasal spray. The openings were sealed with para-film to prevent direct evaporation. The 200-rpm speed was maintained for stirring the receptor compartment. The final sample of volume 0.5 ml was collected by a glass syringe for analysis at 254 nm wavelength of the UV spectrophotometer. To sustain the volume of the sample in the receptor compartment, a fresh pre-heated sample of the same volume was reintroduced. The *in vitro* permeation studies demonstrated that the formulation could increase the time for MF delivery when compared with the commercial nasal spray (Hivate) shown in Figure 7. These results suggest that this system may hold significant potential for drug delivery systems.

**FIGURE 7:** MF release from MSN-MF nano-nasal spray through the silicon membrane compared with the commercial nasal spray.

### 3.10 *In vitro* release study

MF pure drug and formulation MSN-MF was synthesized with the aim to maintain a significant amount of drug release for up to 8 h in order to deliver over-period action. The *in vitro* MF release profile from the MSN-MF showed a biphasic type sustained release pattern, as shown in Figure 8. The pure drug release pattern is very slow in both pH values, which means that MF is basically an insoluble drug (0.00402 mg/ml water solubility). In both media, almost the same pattern of poor solubility is shown. Synthesized formulations showed an initial slow-release pattern of drugs followed by the continual drug release pattern. Due to the presence of the weakly entrapped drug, the initial trend was almost high. Due to slow diffusion and release of drugs from the polymer matrix, a sustained release trend was observed. The fast and burst release of preparation was about 40%–60% in 2 h in acetate buffer with subsequent drug release of 84%–90% in 8 h in 1.2 and 7.4 pH.

**FIGURE 8:** *In vitro* drug release profile of the pure drug and formulation studied at acidic buffer pH 1.2 and phosphate buffer pH 7.4 according to the dialysis bag membrane method (n = 3).

### 3.11 Kinetic modeling

The release of MF from MSN-MF was investigated by using different models on dissolution data: zero order, first order, Korsmeyer–Peppas, and Higuchi. In the present study, MSN-MF was well-suited for the zero-order release model (*R* ^2^ = 0.9419) for up to 8 h (Li et al., 2017). Thus, the remaining mathematical models demonstrated the delivery of the drug incorporated inside the polymeric system after developing the pores through the diffusion mechanism (Dash et al., 2010). The results (Table 1) of *R* ^2^ for the Korsmeyer–Peppas model indicated that MSN-MF followed the super case-2 transport mechanism too, controlled by using the matrix of water absorbency and subsequent relaxation (Treenate and Monvisade, 2017). The following kinetic model was applied to elucidate the release of API through MSN.

**TABLE 1:** Kinetic modeling.

Fitted equations of MSN-MF		
Model	Fitted equation^*^	*R* ^2^
Zero-order	Q = 4.3963t+4.7393	0.97
First-order	Q = -0.1196t+0.0704	0.88
Higuchi	Q = 25.877t^1/2^-22.862	0.93
Korsmeyer–Peppas	Q = 6.63902t^0.85^-2.83593	0.93
Hixson Crowell	(1-Q)^1/3^ = 0.0269t+1.0006	0.92

*In the fitted equations, Q is the accumulated drug released.

### 3.12 Hemolysis investigations

The compatibility of MSN-MF nano-nasal spray with blood was investigated through hemolytic analyses. The results of hemolytic analyses Figure 9 showed that the MSN-MF nano-nasal spray did not cause hemolysis after the administration at concentrations 100, 150, and 200 mg ml^−1^, but negligible hemolysis was noted even at high concentrations, i.e., 200 mg ml^−1^, and the blood cells exhibited significantly considerable tolerance to the complex. The results of the present study demonstrated that cell viability depended upon the concentration, and the cells were alive after incubation with the MSN-MF nano-nasal spray, which confirms blood compatibility.

**FIGURE 9:** Compatibility of the MSN-MF nano-nasal spray with blood.

### 3.13 *In vitro* cell viability testing

According to the results of the MTT assay performed on the human hepatoma cell line (HepG2) over five different concentrations (100, 150, 200, and 400 μg/ml) of MSN-MF nano-nasal spray, the viability of the cell was less at concentration ≥200 μg/ml of MSN-MF nano-nasal spray formulation Figure 10. Apparently, this cell toxicity in the highest concentration is non-significant. The concentration of MSN-MF nano-nasal spray in water is nearly non-toxic and biocompatible. Percentage cell viability was checked at 100, 150, 200, and 400 μg/ml of MSN-MF nano-nasal spray and was found 80.12 ± 5.36, 72.00 ± 2, 69.00 ± 21, and 59.03 ± 8.97 μg/ml, respectively, demonstrating the dose-dependent pattern of cytotoxicity. The IC_50_ of the MSN-MF nano-nasal spray after 24 h of exposure to HepG2 cells was 802.65 μg/ml, that indicated relatively non-toxic nature.

**FIGURE 10:** Percentage toxicity induced at 100, 150, 200, and 400 μg/ML of MSN-MF nano-nasal spray.

### 3.14 Acute toxicity studies

For the acute toxicity study, a total of six alive healthy rats of average weight 200–300 g were selected. Among these six rats, three were placed in a group named as control, while the remaining three rats represented the second group named as the MSN-MF nano-nasal spray group. Nano nasal spray volume equivalent to 10 mg/kg was administered to rats through the nasal passage to MSN-MF group rats. The control group was given water and food. For physical examination of the rats for different parameters, i.e., body weight, clinical findings on the first day and 14th day of the study were noted (Table 2). For biochemical and hematological analysis on the 14th day of the study, 1.0 ml blood was drawn. The results of both biochemistry and hematology are mentioned in Table 2. There was no morbidity and mortality observed in both groups, and hemoglobin, Hct, RBC, and WBC parameters do not show any significant difference when compared to the control group. In spite of some slight differences between the groups, all the hematologic parameters were within normal ranges. Figure 11 shows the images obtained after toxicity evaluation.

**TABLE 2:** Biochemical blood analysis.

Hematology	Group 1	Group 2	Group 3
	MSN-MF	Control	Commercial product
Hb (10–15) g/dl	11.8	12.2	12.8
Hct	41.6	41.8	43.7
WBCs × 10^9^/L	6.1	5.2	6.5
RBCs × 10^6^/mm^3^	5.72	5.76	5.96
Platelets × 10^9^/L	258	286	262
Monocytes (%)	03	07	09
Neutrophils (%)	40	40	52
Lymphocytes (%)	52	50	60
MCV (%)	74.2	72.1	78.2
MCH pg/cell	21.8	18.6	24.4
MCHC (%)	30.4	30.4	31.1
Eosinophils	02	03	02
Blood sugar random mg/dl	71	52	82
Uric acid (serum)mg/dl	8.1	5.76	7.9

**FIGURE 11:** **(A)** Control mouse showing healthy lungs. **(B)** Mouse lung showing resolved inflammation at the peribronchial region. **(C)** Diseased mouse lung showing goblet cell hyperplasia (black circle). **(D)** Diseased mouse lung showing inflammation in alveoli (black circle**)**.

### 3.15 Effect of MSN-MF nano-nasal spray on total inflammatory cells in blood

The results indicate a significant increase in the total leukocyte count of group II (disease) as compared to group I (control) (10.28 ± 1.73 vs. 6.7 ± 1.53). Group III treated with the commercial product showed a significant decrease in MFC as compared to group II (6.52 ± 0.51 vs. 10.28 ± 1.73). There was a significant decrease in MFC of group IV treated with MSN-MF as compared to group II (5.89 ± 0.51 vs. 10.28 ± 1.73) (Table 3).

**TABLE 3:** MSN-MF nano-nasal spray comparison with Hivate.

Formulation	Clarity	pH	Homogeneity	Viscosity (cpi)
MSN-MF nano-nasal spray	Clear	6.8	Good	89
Commercial product	Clear	6.1	Good	67

### 3.16 Effect of MF-MG on IL-4 and IL-5 mRNA expression levels

The results indicate a significant increase in mRNA levels of IL-4 and IL-5 of group II (disease) as compared to group I (control) (6.781 ± 0.117 vs. 5.386 ± 0.189). Group III treated with the commercial product did not show a significant decrease in IL-4 and IL-5 levels as compared to group II (6.604 ± 0.287 vs. 6.781 ± 0.117). However, there was a significant decrease in IL-4 and IL-5 levels of group IV as compared to group II (5.424 ± 0.19 vs. 6.781 ± 0.117) when administered the MSN-MF nano-nasal spray. We have shown forward and reverse sequences in Table 4 for IL-4 and IL-5. The results showed MSN-MF nano-nasal spray when given topically to mice; inflammation significantly decreased eosinophils and neutrophils in the blood as shown in Table 5, and the BALF along with decreasing DTH magnitude. Similarly, a significant decrease in inflammatory cells was observed, when the MF commercial product was applied to mice. Inhibition of mRNA expression of IL-4 may be one of the mechanisms by which MSN-MF nano-nasal spray showed its anti-inflammatory effect. We have mentioned the values of the controlled group and diseased group for compression with our sampled group. We found our sampled group has no significant change as we also went through the previous literature works regarding these values and found satisfactory results.

**TABLE 4:** Cytokine interleukin 4 (IL-4) and cytokine interleukin 5 (IL-5).

Synonym	Cytokine interleukin 4 (IL-4)
Forward sequence	5′-GGC​TGA​AAG​GGG​GAA​AGC​AT-3′
Reverse sequence	5′-CCT​TGC​CGC​CAG​TCT​TTC​AT-3
Synonyms	Cytokines Interleukin 5 (IL-5)
Forward sequence	5-GGA​ATA​GGC​ACA​CTG​GAG​AGT​C-3
Reverse sequence	5-CTC​TCC​GTC​TTT​CTT​CTC​CAC​AC-3

**TABLE 5:** Mean ± SD of MFC and DLC in blood in all groups (n = 6).

Parameter (blood)	Group I (control)	Group II (disease)	Group III commercial product	Group IV MSN-MF nano-nasal spray
MFC 1000/ul	6.7 ± 1.53	10.28 ± 1.73^a^	8.74 ± 1.49 ^b^	6.52 ± 0.51^b^
Lymphocytes (%)	4.7 ± 0.56	5.5 ± 0.1	4.1 ± 0.07	3 ± 0.17
Neutrophils (%)	1.06 ± 0.08	2.3 ± 0.56^a^	1.95 ± 0.22^b^	1.2 ± 0.34
Eosinophils (%)	0.08 ± 0.03	0.57 ± 0.09^a^	0.09 ± 0.05^b^	0.33 ± 0.002^b^
Monocytes (%)	0.23 ± 0.12	0.57 ± 0.01^a^	0.51 ± 0.01	0.49 ± 0.01
Basophils (%)	0.02 ± 0.001	0.03 ± 0.002	0.03 ± 0.001	0.02 ± 0.001

## 4 Discussion

In the medical treatment, CRS topical steroids are the first line of treatment. However, topical steroids frequently have minimal therapeutic effects, mostly because they are poorly distributed to the nose and sinuses (Maurya et al., 2019; Singh et al., 2020b; Far et al., 2020; Singh et al., 2021; Singh et al., 2022). Utilizing the MSN-MF nano-nasal spray for localized drug delivery may improve treatment success by allowing for more consistent administration to desired areas, increased contact duration, increased local drug concentrations, and a reduction in systemic side effects. In order to increase drug absorption, the MSN-MF nano-nasal spray has been utilized as a respiratory drug delivery system. They can reduce mucociliary clearance and prevent macrophage phagocytosis.

## 5 Conclusion

The present study suggested that the MSN-MF nano-nasal spray is a well-optimized formulation for potential treatment of CRS. The *in vitro* studies demonstrated that the following formulation might sustain release for up to 8 h. The *in vitro* MF release from MSN-MF showed initial burst release followed by a sustained release phase. The kinetics of drug release followed anomalous zero-order and Korsmeyer–Peppas and fabricated MSN can also be used for other nasal drug delivery. Thus, the present study provides innovative formulation in intranasal delivery of MSN-MF nano-nasal spray for the treatment of CRS. Minor adaptations in various formulation factors can be fitted for other pharmaceutical usage, and it will be a subject of our future studies. In conclusion, we expect that controlled release of MF using MSN-MF will be a promising approach for improving the local treatment of CRS; hence, their potential for nasal delivery applications warrants further *in vitro* and *in vivo* investigations.

## Data Availability

The original contributions presented in the study are included in the article/Supplementary Material; further inquiries can be directed to the corresponding authors.
